This article has been retracted.

# The Application Value of Clinical Intervention Approaches Based on the Guidance of Knowledge, Belief, and Action Theory for Children with AB and the Analysis of Risk Factors for Poor Prognosis

**DOI:** 10.1155/2023/1816818

**Published:** 2023-02-17

**Authors:** Yuqin Cui, Yu Ni, Haiyan Yan

**Affiliations:** Department of Pediatrics, Yingshang People's Hospital, Fuyang 236000, China

## Abstract

In order to explore the clinical efficacy of knowledge, information, and action theory combined with clinical nursing in children with asthmatic bronchitis (AB) and to analyze the influencing factors of poor prognosis, a total of 98 children with AB in our hospital from January 2021 to August 2022 are collected. The baseline data are analyzed and are randomly divided into a combination group (*n* = 49) and a single group (*n* = 49). The experimental results show that the baseline data of the research subjects are not comparable (*P* > 0.05), the clinical efficacy of the combined group is higher than that of the single group, and the level of pulmonary function indexes in the combined group is significantly higher than that of the single group (*P* < 0.05). The observation shows that family history, repeated respiratory virus infection, and allergy history are all risk factors affecting the prognosis of children with AB.

## 1. Introduction

Asthmatic bronchitis (AB) is common in infants and young children and is a respiratory infectious disease caused by mycoplasma pneumoniae, influenza virus, and respiratory syncytial virus [1]. The common clinical symptoms are mainly cough, wheezing, shortness of breath, etc., and the disease often occurs repeatedly. If there is no timely intervention, some children may even develop bronchial asthma, which has a serious impact on the health and life of the children [2]. At this stage, aerosol absorption is the gold standard for the treatment of the disease, but unlike adults, children will inevitably experience fear and tension in unfamiliar environments, which affects the aerosol treatment [3].

Therefore, appropriate intervention during treatment can better exert the efficacy of nebulization and improve the symptoms of children. The clinical intervention pathway is a holistic nursing program that integrates multiple disciplines, which can have a positive effect on the clinical treatment of children [4]. However, this nursing method still has certain limitations and is not enough to achieve better curative effect. Based on this, this study is guided by the theory of knowledge, belief, and action on the basis of clinical intervention paths to observe the clinical curative effect of the combination of the two nursing methods on children with AB.

The rest of this paper is organized as follows: Section 2 discusses related work, followed by focusing on the observation indicators and statistical methods in Section 3. The pulmonary function and univariate analysis of the influencing factors are discussed in Section 4.  Section 5 concludes the paper.

## 2. Related Work

The theory of knowledge, belief, and action was the most commonly used model to explain the influence and change of personal knowledge and beliefs on health behavior. It could help clients change their health beliefs, build a health knowledge system, and establish health beliefs [5]. Therefore, this theory was applicable to the families of children. In pediatric care, family members were the most important group of medical staff. If family members had one-sided disease awareness, it might lead to poor treatment compliance and affect disease recovery [6]. In this study, clinical intervention was combined with the theoretical model of knowledge, belief, and action. The results showed that the clinical efficacy of the combined group was significantly higher than that of the single group [7]. It showed that the theoretical model of knowledge, belief, and action combined with clinical nursing could not only implement individualized intervention for children but also further deepen family members' cognition of the disease and improve family members' vigilance and enthusiasm for treatment, so as to take correct medication, treat patiently, and speed up the recovery of children.

The repeated episodes of wheezing, shortness of breath, chest tightness, and other phenomena associated with AB disease would lead to changes in lung function, thereby affecting the level of lung function. If not intervened in time, it may lead to hypoxemia and pulmonary hypertension and even lead to severe diseases such as respiratory failure [8]. The use of targeted nursing intervention could significantly improve the level of lung function and coagulation function in children with AB [9]. It showed that clinical nursing combined with the theoretical model of knowledge, belief, and action could significantly improve the level of lung function decline in children. In order to investigate the reason, combined intervention could provide effective health management guidance for children and their families and implement specific respiratory function exercises, which could significantly improve children's lung function [10].

The number of infants and young children with a family history of the risk of AB disease increased [11]. Studies have shown that the incidence of AB in children with recurrent respiratory viral infection was significantly higher than that in children without repeated viral infection [12]. It showed that repeated respiratory virus infection was the influencing factor for inducing AB.

## 3. Observation Indicators and Statistical Methods

The baseline data of 98 children with AB who are diagnosed and treated in our hospital from January 2021 to August 2022 are analyzed, and they are randomly divided into a combined group and a single group. The inclusion criteria are as follows: (1) meet the diagnostic criteria of AB disease, (2) high degree of treatment cooperation, (3) receive glucocorticoid aerosol therapy, (4) complete clinical data, and (5) the family members of the children are informed about the study and sign the consent form. The exclusion criteria are as follows: (1) children with congenital heart disease, (2) children with immunodeficiency and respiratory failure, (3) children with mental disorders and hearing impairments, and (4) unable to participate in this study throughout.

A single group receives clinical interventions as follows: (1) the AB intervention group is set up by professional medical staff to evaluate various indicators of children with AB based on multiparty literature and their own clinical experience. (2) The nursing team members regularly organize knowledge training to consolidate and deepen the content of clinical nursing paths and related treatment methods. At the same time, the team members need to introduce the content and functions of clinical nursing to the families of the children in detail, so as (3) to strengthen the family members' compliance with treatment, provide the corresponding drug care to the child in a timely manner, and, at the same time, inform the family of the child about the knowledge and principles of the drug, instruct the family to pay attention to the relevant precautions, and deal with the adverse reaction in a timely manner and (4) to actively carry out health education and psychological intervention for the families of children, introduce disease-related knowledge, and strengthen family members' understanding of the disease and its intervention effects, thereby reducing family members' negative emotions such as tension and fear and relieving psychological pressure.

The combined group is guided by the combined use of knowledge, belief, and action theory based on a single group intervention. The specific contents are as follows. (1) Understand: collect baseline data such as age, gender, and birth status. At the same time, family-related baseline data (occupation, education level, age, etc.) are collected to preliminarily estimate the family's cognition of the disease and understand its exact needs. Relevant knowledge such as disease etiology, clinical signs, intervention measures, and treatment background is determined. At the same time, an on-site demonstration operation is set up, and the medical staff comments on the operation of the family members, encourages the family members to communicate with each other, and solves the family members' questions. (2) Trust: help family members deal with the problems encountered during the intervention, always pay attention to the psychological state of family members, and provide timely guidance to ensure that family members treat the disease with a positive and correct attitude and build confidence in treatment. (3) Action: instruct family members to pay more attention to their children's diet. The diet structure needs to be healthy and scientific, eating more foods rich in vitamins and proteins that are easy to digest and avoiding cold, irritating, and sweet foods. In addition, the ward should be ventilated in time, maintaining a suitable humidity, ensuring the bed supplies should be replaced in time to reduce virus invasion, and paying attention to scientific medication.

Observation indicators are as follows:

1. The clinical efficacy of the research subjects is analyzed. (1) Significantly effective: 2 days after the intervention, the wheezing and pulmonary wheezing are completely relieved. (2) Effective: 7 days after the intervention, the wheezing and pulmonary wheezing are significantly relieved. (3) Ineffective: Seven days after the intervention, the clinical symptoms of the children did not change or even worsened compared with those before the intervention. Treatment effective rate is equal to (marked number + effective number)/total × 100%
2. Analyze the pulmonary function level of the research subjects, including forced expiratory volume in 1 s (FEV1), forced vital capacity (FVC), and the percentage of FEV1 in FVC (FEV1/FVC%)
3. Univariate analysis of the influencing factors of poor prognosis in children with AB
4. Binary logistic regression analysis of risk factors affecting the prognosis of children with AB

The data are unified and entered into SPSS 26.0 software for processing. The measurement data are expressed as mean ± standard deviation ($\bar{x}\pm s$), the independent sample *t* test is used for the data between groups, and the *F* test is used between multiple groups. The count data are expressed as a percentage (%). Repeated measures analysis of variance is used for comparison of each time period between groups, and spherical test is performed.

## 4. Pulmonary Function and Univariate Analysis of the Influencing Factors

### 4.1. Baseline Data

Table 1 is the analysis of the baseline data of the research subjects. It is clearly evident from Table 1 that the age, gender, length, body weight, course of disease, and other baseline data of the research subjects are not comparable (*P* > 0.05).

### 4.2. Clinical Efficacy of Research Subjects

Table 2 is the analysis of the clinical efficacy of the research subjects after intervention. It is clearly evident from Table 2 that after intervention, the effective rate of the combined group is 91.84%, which is significantly higher than that of the single group.

### 4.3. Pulmonary Function of Subjects before and after Intervention

Table 3 is the analysis of the pulmonary function indexes of the subjects before the intervention and 1 month and 3 months after the intervention. It is clearly evident from Table 3 that before the intervention, the pulmonary function indexes of the research subjects are not comparable.

Figure 1 is the FEV1 levels before and after intervention. It is clearly evident from Figure 1 that the pulmonary function indexes in the 1 and 3 months after the intervention are higher than those before the intervention.

Figure 2 is the FVC levels before and after intervention. It is clearly evident from Figure 2 that the pulmonary function indexes in the combined group are higher than those in the single group after the intervention (*P* < 0.01).

Figure 3 is the FEV1/FVC levels before and after intervention. It is clearly evident from Figure 3 that the pulmonary function indexes in the joint group are higher than those in the single group after the intervention.

### 4.4. Univariate Analysis of the Influencing Factors of Poor Prognosis in Children with AB

Table 4 is the influencing factors of poor prognosis in children with AB by univariate analysis. It is clearly evident from Table 4 that 43 children have poor prognosis and 55 have good prognosis.

### 4.5. Binary Logistic Regression Analysis of Risk Factors Affecting the Prognosis of Children with AB

Table 5 is the variable assignment table. It is clearly evident from Table 5 that the factors contain family history, recurrent respiratory viral infections, allergy history, and prognosis.

Table 6 is the binary logistic regression analysis of risk factors affecting the prognosis of children with AB. It is clearly evident from Table 6 that taking univariate *P* < 0.05 as the independent variable and prognosis as the dependent variable, family history, repeated respiratory virus infection, and history of allergies are independent risk factors for the prognosis of children with AB.

## 5. Conclusion

Family history, repeated respiratory tract infection, and history of allergies are independent risk factors for the prognosis of children with AB. The application of the theory of knowledge, belief, and action combined with clinical intervention can effectively improve the clinical symptoms of children with AB and improve their lung function, and at the same time, it can increase the family members' treatment compliance and enthusiasm, speed up the recovery of children, and improve family members' satisfaction. However, the number of research objects selected in this paper is small and the scope is narrow, and the results may be biased to some extent. Therefore, it is necessary to further increase the number and scope of selected research objects on this basis for further exploration, so as to provide clinical intervention for children with AB.

## Figures and Tables

**Figure 1:** FEV1 levels before and after intervention.

**Figure 2:** FVC levels before and after intervention.

**Figure 3:** FEV1/FVC levels before and after intervention.

**Table 1:** Analysis of baseline data of research subjects ($\bar{x}\pm s$, *n* (%)).

Category	Joint group	Control group	*t*/*x*^2^	*P*
Number of cases	49	49		
Age (months)	16.43 ± 2.89	16.20 ± 3.02	0.647	0.076
Male	24	26	0.761	0.068
Female	25	23		
Length (cm)	81.55 ± 12.79	82.03 ± 12.56	0.325	0.091
Body mass (kg)	13.30 ± 3.57	13.06 ± 3.13	0.477	0.087
Disease duration (d)	5.84 ± 2.04	5.23 ± 1.96	0.924	0.059

**Table 2:** Analysis of the clinical efficacy of the research subjects after intervention (*n* (%)).

Group	Number of cases	Effective	Efficient	Invalid	Efficient
Joint group	49	28 (57.14)	17 (34.69)	4 (8.17)	45 (91.84)
Single group	49	17 (34.69)	19 (38.78)	13 (26.53)	36 (73.47)
*x* ^2^		7.665	7.132	8.574	7.636
*P*		<0.001	<0.001	<0.001	<0.001

**Table 3:** Analysis of the pulmonary function indexes of the subjects before the intervention and 1 month and 3 months after the intervention ($\bar{x}\pm s$).

Group	Time	FEV1 (%)	FVC (L)	FEV1/FVC (%)
Combined group (*n* = 45)	Before intervention	1.22 ± 0.24	2.02 ± 0.24	64.56 ± 5.02
	1 month after intervention	2.13 ± 0.57	2.32 ± 0.68	73.78 ± 4.87
	3 months after intervention	2.98 ± 0.79	3.15 ± 0.26	84.76 ± 5.22

Single group (*n* = 45)	Before intervention	1.24 ± 0.21	2.03 ± 0.13	63.56 ± 5.09
	1 month after intervention	1.67 ± 0.46	2.25 ± 0.54	67.32 ± 4.77
	3 months after intervention	2.03 ± 0.65	2.58 ± 0.46	76.56 ± 4.88

*F* time		152.21	169.15	141.77

*P* time		<0.001	<0.001	<0.001

*F* time point∗group		173.42	138.27	153.86

*P* time point∗group		<0.001	<0.001	<0.001

**Table 4:** Influencing factors of poor prognosis in children with AB by univariate analysis (*n* (%)).

Factor	*n*	Poor prognosis (*n* = 43)	Good prognosis (*n* = 55)	*x* ^2^	*P*
Age (months)					
>12	47	22 (46.81)	25 (53.19)	0.135	0.082
≤12	51	21 (41.18)	30 (58.82)		
Gender					
Male	50	23 (46.00)	27 (54.00)	0.374	0.073
Female	48	20 (41.67)	28 (58.33)		
Height					
Normal	55	25 (45.45)	30 (54.55)	0.381	0.072
Abnormal	43	18 (41.86)	25 (58.14)		
Body mass					
Normal	42	18 (42.86)	24 (57.14)	0.533	0.064
Abnormal	56	25 (44.64)	31 (55.36)		
Family history					
Have	41	27 (65.85)	14 (34.15)	9.872	<0.001
None	57	16 (28.07)	41 (71.93)		
Recurrent respiratory viral infections					
Yes	51	38 (74.51)	13 (25.49)	8.665	<0.001
No	47	6 (12.77)	41 (87.23)		
Allergy history					
Have	45	30 (66.67)	15 (33.33)	8.724	<0.001
None	43	3 (6.98)	40 (93.02)		
Birth status					
Natural delivery	57	25 (43.86)	32 (56.14)	0.773	0.052
Cesarean section	41	18 (43.90)	23 (56.10)		
Feeding method					
Kiss	58	26 (44.83)	32 (55.17)	0.124	0.087
Milk powder	40	17 (42.50)	23 (57.50)		

**Table 5:** Variable assignment table.

Factor	Variable name	Assign
Family history	X1	Yes = 1, no = 2
Recurrent respiratory viral infections	X2	Yes = 1, no = 2
Allergy history	X3	Yes = 1, no = 2
Prognosis	Y	Bad = 1, good = 2

**Table 6:** Binary logistic regression analysis of risk factors affecting the prognosis of children with AB.

Influencing factors	*B*	S.E.	Wald	*P*	OR	95% CI
Have a family history	1.434	1.238	7.576	<0.001	0.117	0.082~0.756
Recurrent respiratory viral infections	1.719	1.108	8.446	<0.001	0.082	0.053~0.606
Have a history of allergies	1.553	1.221	8.764	<0.001	0.089	0.046~0.285

## Data Availability

The simulation experiment data used to support the findings of this study are available from the corresponding author upon request.

## References

[1] Reeves S. R., Barrow K. A., Kolstad T. K. (2018). Fibroblast gene expression following asthmatic bronchial epithelial cell conditioning correlates with epithelial donor lung function and exacerbation history. *Scientific Reports*.

[2] Tian M., Chen M., Bao Y. (2019). Microbial contributions to bronchial asthma occurrence in children: a metagenomic study. *Journal of Cellular Biochemistry*.

[3] Huang J. (2018). Observation and mechanism discussion on budesonide atomization inhalation in the treatment of asthmatic bronchitis in children. *Journal of Clinical Medical Literature*.

[4] Chen G., Xu F., Zhou B. (2021). Effect of comprehensive nursing intervention on the improvement of clinical symptoms and nursing satisfaction of children with febrile convulsion. *Indian Journal of Pharmaceutical Sciences*.

[5] Jing M., Xue J., Kang Y. (2019). Effect of nursing intervention model based on information-knowledge-belief-behavior theory on rehabilitation of patients with gastrointestinal cancer underwent PICC catheterization. *Hainan Medical Journal*.

[6] Ling Z., Hong-wu K. (2019). Effect of continuous nursing intervention based on WeChat platform on post-operative psychological elasticity and shame of breast cancer patients. *Chinese Journal of General Practice*.

[7] Zahiruddin W. M., Arifin W. N., Mohd-Nazri S. (2018). Development and validation of a new knowledge, attitude, belief and practice questionnaire on leptospirosis in Malaysia. *BMC Public Health*.

[8] Nieto A., Mazón A., Nieto M. (2021). Bacterial mucosal immunotherapy with MV130 prevents recurrent wheezing in children: a randomized, double-blind, placebo-controlled clinical trial. *American Journal of Respiratory and Critical Care Medicine*.

[9] Tachimoto H., Imanari E., Mezawa H. (2020). Effect of avoiding cow’s milk formula at birth on prevention of asthma or recurrent wheeze among young children: extended follow-up from the ABC randomized clinical trial. *JAMA Network Open*.

[10] Rocha G. (2021). Inhaled pharmacotherapy for neonates: a narrative review. *Turkish Archives of Pediatrics*.

[11] Chen Y., Xu T. (2018). Association of vitamin D receptor expression with inflammatory changes and prognosis of asthma. *Experimental and Therapeutic Medicine*.

[12] Song Y., Li R. (2021). Effect of budesonide combined with salbutamol nebulization on pulmonary function and serum immune factors in children with bronchiolitis. *American Journal of Translational Research*.

